# Long noncoding RNA HCG11 inhibited growth and invasion in cervical cancer by sponging miR‐942‐5p and targeting GFI1

This article has been retracted.

**DOI:** 10.1002/cam4.3203

**Published:** 2020-08-13

**Authors:** Yan Zhang, Jun Zhang, Lin Mao, Xing Li

**Affiliations:** ^1^ Department of Obstetrics and Gynecology Renmin Hospital of Wuhan University Wuhan China

**Keywords:** cervical cancer, growth, lncRNA HCG11, invasion, miR‐942‐5p

## Abstract

Long noncoding RNAs (lncRNAs) act as essential regulators in cancer tumorigenesis. Our study aimed to explore the underlying mechanism of lncRNA human leukocyte antigen complex group 11 (HCG11) in cervical cancer (CC) progression. Long noncoding RNA HCG11 was downregulated in CC. Functional assays demonstrated that lncRNA HCG11 inhibited CC cell proliferation and invasion. Then, we confirmed that lncRNA HCG11 could directly bind to miR‐942‐5p. Moreover, inhibition of miR‐942‐5p suppressed the growth and invasion of CC cells, and growth factor‐independent transcription repressor 1 (*GFI1*) gene was the target gene of miR‐942‐5p. Long noncoding RNA HCG11 increased the expression of *GFI1* and suppressed cell proliferation and invasion by acting as a miR‐942‐5p sponge. Finally, the overexpression of lncRNA HCG11 suppressed the proliferation and metastasis of CC cells in vivo.

## Graphical abstract

Long noncoding RNA human leukocyte antigen complex group 11 (HCG11) was downregulated in cervical cancer (CC). Long noncoding RNA HCG11 inhibited growth and invasion in CC by sponging miR‐942‐5p and targeting growth factor‐independent transcription repressor 1. The overexpression of lncRNA HCG11 suppressed the proliferation and invasion of CC cells in vivo.

## 1 INTRODUCTION

Cervical cancer (CC) is one of the most common neoplasms of female reproductive organs.^1^, ^2^, ^3^ Even if patients with CC receive the standardized treatment regimen, they are at high risk of recurrence and morbidity.^4^, ^5^ Discovering novel clinical targets and understanding the underlying mechanisms of CC are the cornerstones of creating new treatment strategies.

Long noncoding RNAs (lncRNAs) are noncoding RNA molecules longer than 200 nucleotides.^6^, ^7^, ^8^ Different lncRNAs play various roles in the development of tumor. Long noncoding RNA PLAC2 decreases RPL36 expression by binding with STAT1 and attenuates glioma cell cycle progression.^9^ Long noncoding RNA HOTAIR facilitates gastric cancer cell epithelial mesenchymal transition (EMT) by upregulating histone H3 lysine 27 acetylation.^10^ Long noncoding RNA BLACAT1 increased the viability of cisplatin (DDP)‐resistant cells by downregulating autophagy in non–small cell lung cancer (NSCLC) cell.^11^ Long noncoding RNA human leukocyte antigen complex group 11 (HCG11) acts as a cancer suppressor in several tumors. Long noncoding RNA HCG11 suppresses glioma cell proliferation by sponging miR‐496 and downregulating CPEB3.^12^ Upregulation of lncRNA HCG11 inhibits PI3K/AKT axis and weakens cell invasion in prostate cancer.^13^ However, the role of lncRNA HCG11 in CC is unclear.

MicroRNAs (miRNAs) are small noncoding RNAs of 20‐25 nucleotides in length that downregulate downstream genes by targeting their 3′ untranslated region (UTR).^14^, ^15^ Several researchers demonstrated that competing endogenous RNAs (ceRNAs) have become a vital communication mechanism among lncRNAs and miRNAs. Long noncoding RNAs act as important regulators by sponging miRNAs in various tumors. Downregulation of lncRNA FOXD2‐AS1 suppresses glioma cell invasion by sponging miR‐98‐5p and upregulating CPEB4.^16^ Long noncoding RNA DNM3OS strengthens cell transformation by sponging miR‐29a and miR‐361.^17^ Long noncoding RNA LINC01111 inhibits tumor metastasis by regulating miR‐3924/DUSP1 axis.^18^ Thus, exploring the roles of lncRNAs in CC can help determine potential mechanisms from a new perspective.

This current research indicated that lncRNA HCG11 level was decreased in CC cell lines, thereby suggesting that lncRNA HCG11 might play as a tumor suppressor in CC progression. Gain‐ and loss‐of‐function experiments were performed in vitro and in vivo to investigate the roles and underlying mechanism of lncRNA HCG11. Human leukocyte antigen complex group 11 inhibited growth and invasion in CC by sponging miR‐942‐5p and targeting the growth factor‐independent transcription repressor 1 (*GFI1*) gene.

## 2 MATERIALS AND METHODS

### 2.1 Cell culture

Four human CC cell lines (HeLa, C33A, SiHa, and Caski) and the normal cervical squamous cell line Ect1/E6E7 were cultured in RPMI1640 medium (Gibco) supplemented with 10% fetal bovine serum (Gibco) and incubated at 37°C with 5% CO_2_.

### 2.2 Cell transfection and lentivirus production

Lentiviral vectors for IncRNA HCG11, including LV‐IncRNA HCG11 and sh‐IncRNA HCG11, were purchased from GeneCreate Biological Engineering Co., Ltd. The sequence of GFI1 was cloned into the pcDNA3.1 vector, and the negative control was the empty vector of pcDNA3.1. PcDNA3.1 was purchased from Jing Kairui Biological Engineering. Lipofectamine 3000 (Invitrogen) was applied for transfection following manufacturer's instructions.

### 2.3 Transwell migration and invasion assay

Cervical cancer cells were used for transwell experiment 48 hours after transfection. For the migration assays, transfected cells (N = 4.2 × 10^3^) were plated in top chambers with a noncoated membrane (Gibco). For the invasion assays, transfected cells (N = 6.5‐7.5 × 10^3^) were plated in top chambers with a coated membrane. The number of invading cells was counted after fixing with 4% paraformaldehyde. After 12 hours, crystal violet was used to stain the invading CC cells for counting under a microscope.

### 2.4 Cell counting kit‐8 assay

Cell counting kit‐8 (CCK8) assay was performed following previously described methods.^19^, ^20^ CC cells (N = 2.5 × 10^3^‐3.5 × 10^3^) were seeded in 96‐well plates 48 hours after transfection. Six holes were considered one group. Cell counting kit‐8 (60‐80 μL, Beyotime) was added into every hole 1 hour before detection. Microplate reader was used to determine the optical density every 12 hours at 450 nm.

### 2.5 RNA sample preparation

RNA sample preparation was performed following previously described methods.^21^ Total RNA of CC cells was extracted by TRIzol reagent (Invitrogen) following manufacturer's instructions. The yield and purity of the cell RNA were up to the standard: Abs260/Abs280>1.8.

### 2.6 Quantitative reverse transcription PCR

Total RNA (2‐3 μg) was subjected to quantitative real‐time polymerase chain reaction (qRT‐PCR) according to the manufacturer's instructions. SYBR Green qPCR Master Mix (Takara) was used to detect the miRNA expression level. Growth factor‐independent transcription repressor 1 and GAPDH expression levels were examined using the following specific primers: 5′CCGCGCTCATTTCTCGTCA3′; 5′ACGGAGGGAATAGTCTGGTCC3′; 5′GGAGCGAGATCCCTCCAAAAT3′ and 5′GGCTGTTGTCATACTTCTCATGG3′.

The 2^−ΔΔCt^ method was used to calculate the expression level‐fold changes of genes.

### 2.7 Luciferase reporter assay

Luciferase reporter assay was carried out as described in the literature.^22^, ^23^ Specific binding sites between IncRNA HCG11 and miR‐942‐5p and between miR‐942‐5p and GFI1 were predicted by StarBase and Targetscan. Wt‐pmirGLO‐IncRNA HCG11, Wt‐pmirGLO‐GFI1, and mut‐pmirGLO (knockdown combination between IncRNA HCG11 and miR‐942‐5p and between miR‐942‐5p and GFI1) were constructed. Wt‐pmirGLO or mut‐pmirGLO was transfected into CC cells with mimic/inhibitor‐942‐5p. Finally, the luciferase activity of every group was normalized to the total protein concentration of CC cells.

### 2.8 In vivo study

Female nude mice (6 weeks old) were purchased from Laboratory Animal Center. A IncRNA HCG11‐stable overexpression SiHa cell line was constructed. Xenograft tumor models were established by subcutaneous transplantation. For the xenograft tumor model, 6 × 10^6^ cells were subcutaneously injected into the left inguinal area of nude mice. The volume of xenograft tumors was counted at 0, 5, 10, 15, 20, and 25 days. The weight of xenograft tumors was obtained after 25 days. Lung metastasis mouse model was also established through intrasplenic injection of 4.5 × 10^6^ SiHa cells stably overexpressing IncRNA HCG11 or LV‐NC. Lung colonization capacity was evaluated after 25 days. The number of lung metastatic foci was counted after hematoxylin and eosin staining. All animal experiments received approval from the Institutional Animal Care and Use Committee of Our Hospital.

### 2.9 Statistical analysis

GraphPad Prism 6.0 and SPSS 13.0 were used to analyze data. Statistical data were expressed as mean ± SD. Differences were considered significant at *P* < .05.

## 3 RESULTS

### 3.1 Expression level of was downregulated in CC cell lines and suppressed cell invasion and proliferation

IncRNA HCG11 expression level was detected in CC lines. IncRNA HCG11 expression was measured by quantitative reverse transcription PCR (qPCR) in CC cell lines, namely, HeLa, C33A, SiHa, and Caski, and compared with that in normal cervical squamous cell line Ect1/E6E7. IncRNA HCG11 expression level was downregulated in CC cell lines (Figure 1A). Then, overexpression and knockdown of IncRNA HCG11 were performed in HeLa and SiHa. The efficiencies of LV‐IncRNA HCG11 and sh‐IncRNA HCG11 were determined by qPCR. As shown in Figure 1B and C, IncRNA HCG11 expression level was effectively upregulated by LV‐IncRNA HCG11 and downregulated by sh‐IncRNA HCG11. Then, the role of IncRNA HCG11 in cell proliferation was investigated. Cell counting kit‐8 assays indicated that LV‐IncRNA HCG11 suppressed cell growth, whereas sh‐IncRNA HCG11 promoted cell growth in HeLa and SiHa (Figure 1D,E). Moreover, colony formation assays showed that the number of colonies was decreased by LV‐IncRNA HCG11 but increased by sh‐IncRNA HCG11 in CC cells (Figure 1F,G). Transwell migration and invasion assays were performed in HeLa and SiHa. LV‐IncRNA HCG11 weakened cell migration, whereas sh‐IncRNA HCG11 enhanced cell migration in CC cells (Figure 1H,I). Moreover, LV‐IncRNA HCG11 suppressed cell invasion, whereas sh‐IncRNA HCG11 contributed to cell invasion in HeLa and SiHa (Figure 1J,K). Thus, IncRNA HCG11 inhibited the cell growth, migration, and invasion in CC cells.

**FIGURE 1:** IncRNA HCG11 was decreased in cervical cancer cell lines and inhibited cell invasion and proliferation. A, Expression levels of IncRNA HCG11 in cervical cancer cell lines. B and C, The efficiencies of LV‐IncRNA HCG11 and sh‐IncRNA HCG11 were determined through quantitative real‐time polymerase chain reaction in Hela and SiHa. D and E, Cell proliferation of cervical cancer cells were measured using Cell counting kit‐8 assay. F and G, Cell proliferation of cervical cancer cells were measured using colony formation. H and I, Cervical cancer cell migration was inhibited by IncRNA HCG11 overexpression but was enhanced by IncRNA HCG11 knockdown. J and K, Cervical cancer cell invasion was inhibited by IncRNA HCG11 overexpression but was enhanced by IncRNA HCG11 knockdown. The data are representative of three independent experiments. Data are presented as mean ± SD. **P < .01, ***P < .001

### 3.2 MiR‐942‐5p was predicted as the direct target of IncRNA HCG11

Cytoplasmic lncRNA can function as ceRNA.^24^, ^25^ The distribution of IncRNA HCG11 was initially identified in CC cells. qPCR showed that IncRNA HCG11 was chiefly expressed in the cytoplasm of HeLa and SiHa (Figure 2A,B). Fluorescence in situ hybridization assays also revealed that IncRNA HCG11 was mainly localized in the cytoplasm of CC cell (Figure 2C). Four candidate miRNAs, namely, miR‐144‐3p, miR‐155‐5p, miR‐942‐5p, and miR‐1278, were chosen as target miRNAs of IncRNA HCG11 through StarBase (http://starbase.sysu.edu.cn). The candidate miRNAs were screened by qPCR in CC cells transfected with LV‐IncRNA HCG11. Among the four candidates, the expression level of miR‐942‐5p got the largest reduction compared with the negative control after transfection with LV‐IncRNA HCG11. (Figure 2D,E). Moreover, qPCR results indicated that sh‐IncRNA HCG11 upregulated the expression level of miR‐942‐5p in HeLa and SiHa (Figure 2F,G). As shown in Figure 2H and I, IncRNA HCG11 in cell lysis was enriched by a IncRNA HCG11‐specific probe. MiR‐942‐5p cell lysis could be enriched by the IncRNA HCG11‐specific probe (Figure 2J,K). Then, biotin‐coupled miR‐942‐5p captured a fold change of IncRNA HCG11 in the complex as compared with biotin‐coupled NC in CC cells (Figure 2L,M). The specific binding sites between IncRNA HCG11 and miR‐942‐5p were predicted by StarBase v2.0, as shown in Figure 2N. As shown in Figure 2O and P, luciferase activity could be suppressed by mimic‐miR‐942‐5p but enhanced by inhibitor‐miR‐942‐5p in WT‐IncRNA HCG11 reporter. However, the mutant‐type reporter gene (mut‐IncRNA HCG11 reporter) was not inhibited or improved in the luciferase activity by mimic‐ or inhibitor‐miR‐942‐5p. Therefore, miR‐942‐5p was the direct target of IncRNA HCG11.

**FIGURE 2:** miR‐942‐5p was predicted as a direct target of IncRNA HCG11. A and B, qPCR results indicated that IncRNA HCG11 was mainly expressed in the cytoplasm of Hela and SiHa cells. C, Fluorescence in situ hybridization assays results showed that IncRNA HCG11 was mainly located in the cytoplasm. D and E, Four candidate miRNAs were screened by qPCR in cells transfected with LV‐IncRNA HCG11. F and G, The expression level of miR‐942‐5p was upregulated in Hela and SiHa cells transfected with sh‐IncRNA HCG11. H and I, IncRNA HCG11 in cell lysis was pulled down and enriched with IncRNA HCG11‐specific probe and then detected by qPCR. J and K, miR‐942‐5p was pulled down and enriched with IncRNA HCG11‐specific probe and then detected by qPCR. L and M, Biotin‐coupled miR‐942‐5p captured a fold change of IncRNA HCG11 in the complex as compared with biotin‐coupled NC in biotin‐coupled miRNA capture. N, The direct binding sites between IncRNA HCG11 and miR‐942‐5p were presented. O and P, Luciferase reporter assay was performed to confirm the direct binding relationship between IncRNA HCG11 and miR‐942‐5p. In all panels, the data are representative of three independent experiments. Data are presented as mean ± SD. *P < .05, **P < .01, ***P < .001

### 3.3 Effects of miR‐942‐5p on the growth and invasion of CC cells

The efficiency of mimic‐ or inhibitor‐miR‐942‐5p was determined by qPCR in HeLa and SiHa. The miR‐942‐5p expression level was effectively upregulated by mimic‐miR‐942‐5p and was effectively downregulated by inhibitor‐miR‐942‐5p (Figure 3A‐D). Then, the effect of miR‐942‐5p on proliferation was determined by Cell counting kit‐8 assay (CCK8) assays. The mimic‐miR‐942‐5p enhanced cell proliferation in HeLa and SiHa, whereas inhibitor‐miR‐942‐5p suppressed it (Figure 3E‐H). Moreover, transwell assays were performed. The mimic‐miR‐942‐5p promoted cell invasion, whereas inhibitor‐miR‐942‐5p inhibited cell invasion in CC cells (Figure 3I‐L). miR‐942‐5p enhanced the growth and invasion of CC cells.

**FIGURE 3:** Effects of miR‐942‐5p on the growth and invasion of cervical cancer cells. A‐D, The efficiency of mimic‐ and inhibitor‐miR‐942‐5p was determined by qPCR in Hela and SiHa. E‐H, Cell counting kit‐8 assays indicated that mimic‐miR‐942‐5p enhanced but inhibitor‐miR‐942‐5p suppressed cervical cancer cell proliferation. I‐L, Transwell assays results showed that mimic‐miR‐942‐5p promoted but inhibitor‐miR‐942‐5p inhibited cervical cancer cell migration and invasion. In all panels, the data are representative of three independent experiments. Data are presented as mean ± SD. **P < .01, ***P < .001

### 3.4 *GFI1* was the direct target gene of miR‐942‐5p

Four candidate genes, namely, *ZNF23*, *CIR1*, *MCFD2*, and *GFI1*, were chosen as target genes of miR‐942‐5p through Targetscan (http://www.targetscan.org). These candidate genes were screened in HeLa and SiHa transfected with mimic‐miR‐942‐5p. Among the four target genes, the expression level of GFI1 got the largest reduction compared with the negative control after transfection with mimic‐miR‐942‐5p (Figure 4A,B). Moreover, qPCR results indicated that inhibitor‐miR‐942‐5p upregulated the expression level of *GFI1* in CC cells (Figure 4C,D). Moreover, western blot results showed that mimic‐miR‐942‐5p decreased the protein level of GFI1, whereas inhibitor‐miR‐942‐5p increased the expression level of GFI1 (Figure 4E,F). Then, the specific binding sites between miR‐942‐5p and GFI1 were shown in Figure 4G predicted by Targetscan. As shown in Figure 4H and I, luciferase activity could be suppressed by mimic‐miR‐942‐5p but enhanced by inhibitor‐miR‐942‐5p in WT‐GFI1 reporter. However, the mutant‐type reporter gene (mut‐GFI1 reporter) was not inhibited or improved in the luciferase activity by mimic‐ or inhibitor‐miR‐942‐5p. Thus, *GFI1* was a direct target gene of miR‐942‐5p.

**FIGURE 4:** Growth factor‐independent transcription repressor 1 (GFI1) was a direct target gene of miR‐942‐5p. A and B, Four candidate genes were screened by qPCR in cells transfected with mimic‐miR‐942‐5p in Hela and SiHa. C and D, qPCR results indicated that the expression level of GFI1 was upregulated in Hela and SiHa transfected with inhibitor‐miR‐942‐5p. E and F, Western blot showed that the expression level of GFI1 was downregulated by mimic‐miR‐942‐5p but was upregulated by inhibitor‐miR‐942‐5p. G, The direct binding sites between miR‐942‐5p and GFI1 are presented. H and I, Luciferase reporter assay was performed to confirm the direct binding relationship between miR‐942‐5p and GFI1. In all panels, the data are representative of three independent experiments. Data are presented as mean ± SD. **P < .01, ***P < .001

### 3.5 IncRNA HCG11 upregulated the expression level of GFI1 and acted as antioncogene by sponging miR‐942‐5p

The relationship between IncRNA HCG11 and GFI1 was investigated. qPCR and western blot results indicated that IncRNA HCG11 overexpression upregulated the GFI1 expression level, but the knockdown of IncRNA HCG11 downregulated it (Figure 5A‐D). Moreover, the binding sites of miR‐942‐5p and GFI1 were knocked out, and mut‐GFI1 reporter was established. Luciferase reporter assay results indicated that luciferase activity could be upregulated by LV‐IncRNA HCG11 but downregulated by sh‐IncRNA HCG11 in the WT‐GFI1 reporter. However, the mutant‐type reporter gene (mut‐GFI1 reporter) was not inhibited or improved in the luciferase activity by LV‐IncRNA HCG11 or sh‐IncRNA HCG11 (Figure 5E,F). Then, the effect of GFI1 on CC cell growth and invasion was investigated. The efficiency of pcDNA3.1‐GFI1 was determined by qPCR. qPCR and western blot results showed that the expression level of GFI1 was effectively upregulated by pcDNA3.1‐GFI1 in HeLa and SiHa (Figure 5G‐J). Cell counting kit‐8 assay results indicated that overexpression of GFI1 suppressed CC cell growth (Figure 5K,L). Moreover, transwell invasion assays were performed in HeLa and SiHa. Growth factor‐independent transcription repressor 1 overexpression inhibited the CC cell invasion (Figure 5M,N). Furtherly, restore experiments were performed in HeLa and SiHa, and the cells were cotransfected with LV‐IncRNA HCG11 or mimic‐miR‐942‐5p. As shown in Figure 5O and P, mimic‐miR‐942‐5p could restore the inhibition of cell growth after transfection with LV‐IncRNA HCG11. Moreover, mimic‐miR‐942‐5p could restore the inhibition of cell invasion after transfection with LV‐IncRNA HCG11 in HeLa and SiHa (Figure 5Q,R). The IncRNA HCG11 upregulated the expression level of GFI1 and inhibited CC cell growth and invasion by sponging miR‐942‐5p.

**FIGURE 5:** IncRNA HCG11 functions as antioncogene by acting as miR‐942‐5p sponge. A‐D, qPCR and western blot results indicated that the expression level of growth factor‐independent transcription repressor 1 (GFI1) was upregulated by LV‐IncRNA HCG11 but was downregulated by sh‐IncRNA HCG11. E and F, The mutant‐type reporter gene (Mut‐GFI1 reporter) was established, which binds sites of miR‐942‐5p and GFI1 was knockdown. Luciferase reporter assay was performed to confirm the relationship between IncRNA HCG11 and GFI1. G‐J, The efficiency of pcDNA3.1‐GFI1 was determined by qPCR and western blot. K and L, GFI1 overexpression suppressed the growth of cervical cancer cell. M and N, GFI1 overexpression inhibited cell invasion in Hela and SiHa. O and P Cell counting kit‐8 assays were performed in Hela and SiHa. Cells were transfected with LV‐IncRNA HCG11 or mimic‐miR‐942‐5p. Q and R, Transwell assays were performed in cervical cancer cells transfected with LV‐IncRNA HCG11 or mimic‐miR‐942‐5p. In all panels, the data are representative of three independent experiments. Data are presented as mean ± SD.*P < .05, **P < .01

### 3.6 IncRNA HCG11 suppressed CC growth and metastasis in vivo

The xenograft tumor models of CC were constructed by using SiHa cells infected with IncRNA HCG11 lentivirus (every group = 5). A picture of the xenograft is shown in Figure 6A. Then, the efficiency of LV‐IncRNA HCG11 in the xenograft tumor model was determined by qPCR. IncRNA HCG11 was effectively upregulated in the LV‐IncRNA HCG11 group (Figure 6B). The sizes of the xenograft in the LV‐IncRNA HCG11 and LV‐NC groups were calculated every 5 days. The IncRNA HCG11 overexpression suppressed tumor proliferation in vivo (Figure 6C). The weight of the xenografts was calculated. The LV‐IncRNA HCG11 group was significantly lighter than the LV‐NC group (Figure 6D). Lung metastasis models were established by inoculation of SiHa cells. As shown in Figure 6E, IncRNA HCG11 overexpression suppressed the metastasis ability of SiHa cells. Furthermore, the Ki67 expression level was determined in LV‐IncRNA HCG11 and LV‐NC groups. qPCR and western blot results indicated that the Ki67 expression level was downregulated in the LV‐IncRNA HCG11 group (Figure 6F,G). Moreover, the miR‐942‐5p/GFI1 axis was determined. The expression level of miR‐942‐5p was downregulated, whereas that of GFI1 was upregulated in the LV‐IncRNA HCG11 group (Figure 6H‐J). Immunohistochemistry assays also showed that the GFI1 expression level was increased in the LV‐IncRNA HCG11 group (Figure 6K). IncRNA HCG11 suppressed CC growth and metastasis in vivo.

**FIGURE 6:** IncRNA HCG11 suppressed the cervical cancer growth and metastasis in vivo. A, The cervical cancer mouse model was constructed by using SiHa cells infected with LV‐IncRNA HCG11 lentivirus. B, The efficiency of LV‐IncRNA HCG11 in mouse model was determined by qPCR. C, The size of local tumors in these two groups was calculated (n = 5). D, The weight of tumors in these two groups was calculated (n = 5). E, Typical pictures for lung metastasis of mouse model. The percentage of mice with or without metastatic nodules in the lungs was counted. F and G, The expression level of Ki67 was downregulated in LV‐IncRNA HCG11 group. H, The expression level of miR‐942‐5p was downregulated in LV‐IncRNA HCG11 group. I and J, The expression level of growth factor‐independent transcription repressor 1 (GFI1) was upregulated in LV‐IncRNA HCG11 group. K, immunohistochemistry (IHC) assays indicated that the expression level of GFI1 was increased in LV‐IncRNA HCG11 group. In all panels, the data are representative of three independent experiments. Data are presented as mean ± SD. **P < .01, ***P < .001

## 4 DISCUSSION

In this study, lncRNA HCG11 expression level was decreased in CC cell lines. IncRNA HCG11 plays an antioncogene role in glioma and prostate cancer.^12^, ^13^ However, the role of IncRNA HCG11 in CC is unknown. Gain‐of‐function and loss‐of‐function experiments were performed in CC cells. IncRNA HCG11 suppressed cell growth and invasion in HeLa and SiHa. Long noncoding RNAs act as cancer‐promoting or cancer‐suppressing regulator in tumor by acting as ceRNAs.^26^, ^27^ Competing endogenous RNA‐acting lncRNAs regulate coding genes via sharing miRNA binding elements, which set up a posttranscriptional regulatory network.^28^, ^29^ Thus, we are working on the assumption that IncRNA HCG11 inhibited CC progression through ceRNAs. Fluorescence in situ hybridization assays revealed that IncRNA HCG11 was mainly localized in the cytoplasm of CC cell. Luciferase reporter assay results indicated that IncRNA HCG11 played its function as a ceRNA that competitively sponge miR‐942‐5p.

MiR‐942 was identified as an important regulator in tumor. The overexpression of miR‐942 enhances hepatocellular carcinoma cell metastasis by targeting RRM2B.^30^ Overexpression of miR‐942 promotes NSCLC progression by regulating EMT.^31^ We performed gain‐of‐function and loss‐of‐function experiments, and results showed that inhibition of miR‐942‐5p suppressed CC cell growth and invasion. MicroRNA serves its function as a regulator that targets the 3′ UTR of genes.^32^, ^33^ Growth factor‐independent transcription repressor 1 was identified as the direct target gene of miR‐942‐5p. The expression level of *GFI1* is downregulated in cancer cells and suppressed in various cancers. Growth factor‐independent transcription repressor 1 suppresses cell proliferation and invasion in colorectal cancer and oral cancer.^19^, ^34^ Our finding indicated that *GFI1* overexpression suppressed CC cell growth and invasion. Moreover, IncRNA HCG11 upregulated *GFI1* expression level by sponging miR‐942‐5p. Furthermore, the key role of miR‐942‐5p in the function of IncRNA HCG11 was explored. Moreover, restore experiments were performed in HeLa and SiHa. Overexpression of miR‐942‐5p could restore the inhibition of CC cell growth and invasion after transfection with LV‐IncRNA HCG11. Finally, the xenograft tumor model and lung metastasis model were constructed. IncRNA HCG11 suppressed CC cell growth and metastasis in vivo. Moreover, IncRNA HCG11 downregulated miR‐942‐5p and upregulated the *GFI1* expression level in vivo.

In summary, IncRNA HCG11 competitively binds miR‐942‐5p to abolish the inhibitor effect of miR‐942‐5p on GFI1. Gain‐of‐function and loss‐of‐function experiments indicated that IncRNA HCG11 inhibited the growth and invasion of CC cells by sponging miR‐942‐5p and targeting GFI1. Our study provided insights into the role of IncRNA HCG11 in CC progression and its use as a potential therapeutic target for CC.

## CONFLICT OF INTEREST

The authors declare that they have no competing interests.

## AUTHORS' CONTRIBUTIONS

Yan Zhang, Xing Li, and Jun Zhang contributed to the experimental work, figures, and drafting of the manuscript. Yan Zhang and Xing Li designed the study and did data analysis. Lin Mao assisted with the experiments and data analysis. All authors have read and approved the final manuscript.

## ETHICAL APPROVAL

All animal experiments received approval from the Institutional Animal Care and Use Committee of Renmin Hospital of Wuhan University.

## Data Availability

The data and materials used in the present study are available.
